This article has been retracted.

# Effects of Collagen Antibacterial Functional Dressing plus Continuous Nursing on Lower Extremity Skin Injury Caused by Norepinephrine in Patients with Septic Shock

**DOI:** 10.1155/2022/4160637

**Published:** 2022-08-18

**Authors:** Xiaoxia Hu, Hongxia Wang, Yun Lin

**Affiliations:** ^1^Intensive Care Unit, The Third People's Hospital of Hubei Province, Wuhan 430030, China; ^2^Department of Neurology, The Third People's Hospital of Hubei Province, Wuhan 430030, China

## Abstract

**Background:**

This study was designed to explore the effects of collagen antibacterial functional dressing plus continuous care on norepinephrine-induced lower extremity skin injury in patients with septic shock.

**Methods:**

In this prospective, randomized, controlled study, 120 patients with septic shock receiving norepinephrine in our hospital from February 2020 to February 2021 were recruited. All the enrollments were randomized into the experimental group (*n* = 60) and the control group (*n* = 60). The control group received continuous care, while the experimental group additionally received collagen antibacterial functional dressing. Outcome measures included skin sensation scores, incidence of lower extremity skin injuries, recovery time, inflammatory factor levels, and care satisfaction.

**Results:**

Collagen antibacterial functional dressing plus continuous care resulted in significantly lower skin sensation scores and a lower incidence of skin injuries versus continuous care alone. Patients in the experimental group had faster recovery of lower extremity skin injury than those in the control group. Collagen antibacterial functional dressing plus continuous care was associated with significantly lower levels of inflammatory factors and a higher satisfaction rate than continuous care alone.

**Conclusion:**

Collagen antibacterial functional dressing plus continuous care improves the local skin condition of patients with septic shock receiving norepinephrine, regulates the levels of inflammatory factors, reduces the risk of skin injuries, and enhances care satisfaction.

## 1. Introduction

Septic shock is a clinical syndrome characterized by systemic infection. Metabolic disorders and dysfunctions are frequently seen in most cases, in which the hemodynamic effects, inflammatory factors, and immune factors are mutually influenced, leading to homeostasis imbalance or even multiple organ failure in severe cases. The total mortality rate of septic shock ranges from 40% to 70% [1–3]. In current practice, liquid resuscitation plus vasoactive drugs is a well-recognized protocol for septic shock management. Norepinephrine is a commonly used vasoactive drug in clinical practice [4, 5] that regulates the blood pressure of patients, improves their organ perfusion, and prevents organ functional failure; however, it is highly irritating and may cause skin tissue injuries. Mild injury symptoms include redness, pain, and local tissue necrosis, while severe cases may suffer dysfunction, seriously compromising the treatment effect and the nurse-patient relationship [6, 7]. To this end, comprehensive nursing has been identified for complication prevention of the lower extremities to potentiate the efficacy of norepinephrine; nonetheless, the expected treatment outcome is somehow compromised [8, 9]. Previous studies have found that in the treatment of the skin radiation injury of breast cancer patients during radiotherapy [10, 11], the collagen antibacterial functional dressing accelerated cell metabolism, promoted wound healing, relieved skin pain, and regulated the level of local inflammatory factors, which is conducive to injured skin repair. Accordingly, this study was designed to explore the effectiveness of collagen antibacterial functional dressing plus continuous care on the skin injury of lower extremities caused by norepinephrine in patients with septic shock.

## 2. Materials and Methods

### 2.1. General Materials

In this prospective, randomized, controlled study, 120 patients with septic shock treated with norepinephrine in our hospital from February 2020 to February 2021 were included. All the enrollments were randomized into the experimental group (*n* = 60) and the control group (*n* = 60). This study was approved by the ethical committee of our hospital (No. 2020-15/254).

### 2.2. Inclusion and Exclusion Criteria

#### 2.2.1. Inclusion Criteria

Inclusion criteria were as follows: (1) patients or their family members were fully informed of the research process and signed the consent form and (2) patients met the diagnostic criteria for septic shock [12] and were treated with norepinephrine.

#### 2.2.2. Exclusion Criteria

Exclusion criteria were as follows: (1) patients with mental problems that prevented normal communication [13]; (2) patients with other organic diseases [14]; and (3) norepinephrine was not included in the treatment plan.

#### 2.2.3. Withdrawal Criteria

Withdrawal criteria were as follows: (1) patients with adverse events or serious adverse events; (2) patients with disease deterioration during the experiment; and (3) patients who revoked their consent.

### 2.3. Methods

#### 2.3.1. Norepinephrine Therapy

Both groups of patients received an intravenous infusion of norepinephrine (GrandPharma China Co., Ltd., National Medicine Standard H42021301) at the medial malleolus saphenous vein of the lower limbs. The infusion site was altered accordingly in the event of skin injury, and 0.25% procaine was given (Jiangsu Jiuxu Pharmaceutical Co., Ltd., National Medicine Standard H20023101) for partial pain alleviation.

#### 2.3.2. Continuous Care

Both groups of patients were given continuous care. (1) A continuous care exchange group consisting of septic shock patients was established, with the head nurse as the group administrator, and chief physicians were invited to assist the group administration. A continuous care nursing team with two chief physicians, three nurses, a psychologist, and a nutritionist was established to answer the patients' questions and formulate tailored continuous care protocols. The patients and their families were fully informed of the purpose, process, and significance of the study to ensure proactive and effective participation. (2) The patients in the exchange group were named “Department + Patient Name + Bed Number,” which is convenient for information collection and condition monitoring and documentation. Before discharge, the patients were given disease and care instructions, including knowledge of treatment, nursing, and related complications, and were instructed to correctly perform home care. The following conditions during treatment were documented: ① sudden increase or decrease of body temperature; ② impaired consciousness, such as apathy and lethargy; ③ excessive blood pressure fluctuation (an alteration of blood pressure by 15% was considered an excessive fluctuation); and ④ decreased urine output. (3) The patients were informed of the importance of skin management. Patients with septic shock might have flush or clammy skin or have a vascular endometrial injury due to injections of norepinephrine and other drugs, which caused local skin swelling and bruising. (4) Cured cases and proper psychological guidance were introduced to patients to enhance their treatment compliance. (5) The patients were followed up by telephone 3 days after discharge. Then, the telephone follow-up was conducted every 1 month. The duration of follow-up was 3 months.

#### 2.3.3. Collagen Antibacterial Functional Dressing Treatment

The experimental group received collagen antibacterial functional dressing (Tibet Beizhuya Pharmaceutical Co., Ltd., Tibet Naqu Medical Device (2015) No. 1640001) at the norepinephrine injection site. After the injection, with the patients in a sitting position, their skin was cleaned with 37°C water, and the collagen antibacterial dressing was evenly applied to the injection area with a thickness of around 2 mm–3 mm and a diameter of 4 cm around the needlepoint. The dressing was applied once a day before bed. After discharge, the patients were instructed to perform collagen antibacterial functional dressing 3 days later.

### 2.4. Outcome Measures

#### 2.4.1. Skin Sensation Score

The evaluation is based on the skin toxicity assessment tool [15], and the scale includes three domains of treatment characteristics, skin reaction, and patient sensation. There are four items in patient sensation, including burning, itching, pressing pain, and stretching. The Riggett five-level scoring method was adopted to investigate the skin sensation scores of patients before and one month after discharge. The higher the score, the more severe the skin injury.

#### 2.4.2. Incidence of Lower Extremity Skin Injury

The drug extravasation and tissue injury during the treatment of patients were meticulously documented. Mild injury includes skin redness, swelling, subcutaneous induration, and pain in the local exudation area, and severe injury includes local tissue necrosis and dysfunction. The number of patients with skin injuries of lower extremities was recorded to calculate the corresponding incidence.

#### 2.4.3. Recovery Time of Lower Extremity Skin Injury

The recovery time of the patient's lower extremity skin injury was recorded.

#### 2.4.4. Inflammatory Factor Level

5 ml of morning fasting venous blood was collected from the patients before treatment and 1 month after discharge, and the immunoturbidimetric method was used (kit: Nanjing Getein Biotech Co., Ltd., Su Food and Drug Administration Approval Number 2012 No. 2400146) to determine the levels of C-reactive protein (CRP), serum procalcitonin (PCT), and tumor necrosis factor-alpha (TNF-*α*), and the operation process was carried out in strict accordance with the kit instructions.

#### 2.4.5. Care Satisfaction

The hospital's self-developed scale was used to evaluate patients' care satisfaction. The scale has a maximum score of 5 points, with 5 points for highly satisfied, 3-4 points for satisfied, and 2 points and below for dissatisfied. The satisfaction rate 1 month after discharge was calculated.

### 2.5. Statistical Analysis

The selected data processing software for this study was SPSS 20.0, and the graphics were plotted by using GraphPad Prism 7 (GraphPad Software, San Diego, USA). The research included count data and measurement data. The count data were analyzed by the chi-square test, and the measurement data were analyzed by the *t*-test. *P* < 0.05 indicates that the difference is statistically significant.

## 3. Results

### 3.1. Patient Characteristics

The patient characteristics of the two groups were comparable (*P* > 0.05) (Table 1).

### 3.2. Comparison of Skin Sensation Scores of Patients

Collagen antibacterial functional dressing plus continuous care resulted in significantly lower skin sensation scores versus continuous care alone (*P* < 0.001), as shown in Table 2.

### 3.3. Comparison of the Incidence Rate of Skin Injury of the Lower Extremities

A lower incidence of lower limb skin injury in the experimental group was observed (*P* < 0.05), as shown in Table 3.

### 3.4. Comparison of Recovery Time of Patients with Lower Extremity Skin Injury

Patients in the experimental group had faster recovery of lower extremity skin injury than those in the control group (*P* < 0.001) (Figure 1).

### 3.5. Comparison of Inflammatory Factor Levels in Patients

Collagen antibacterial functional dressing plus continuous care was associated with significantly lower levels of inflammatory factors than continuous care alone (*P* < 0.05) (Table 4).

### 3.6. Comparison of Patient Care Satisfaction

A higher nursing satisfaction was obtained in the patients in the experimental group versus the control group (*P* < 0.05) (Table 5).

## 4. Discussion

The results showed that the skin sensation scores and the incidence rate of skin injuries of the experimental group were significantly lower than those of the control group. Pathogenic microorganisms and cell wall products invading the blood circulation during septic shock result in activation of cellular and the humoral immune system, and various endogenous mediators act in the organs and systems, leading to metabolic disorders and even multiple organ failure [16]. In the pathogenesis of septic shock, inflammatory factors are the most important factors that induce hemodynamic alterations and may lead to systemic vasodilation [17] and reduced organ perfusion. Therefore, proper hemodynamic management is key to avoid multiple organ failures [18]. At present, vasoactive drugs are administered for tissue perfusion restoration [19], in which norepinephrine is the most common one for septic shock. Norepinephrine effectively constricts blood vessels, increases arterial blood pressure, and averts internal organ injury. However, norepinephrine has strong penetrability and is prone to drug extravasation, causing vascular smooth muscle spasm, vascular intima damage, and endometritis [20]. Previously, comprehensive care has been recommended for septic shock management to avoid complications secondary to norepinephrine [21] but failed to achieve the expected outcome. In the present study, the incidence of lower extremity skin injury in the experimental group was significantly lower than that in the control group, which may be attributed to the intense antibacterial effects of collagen stock solution, hydrogel, and polylysine in the collagen antibacterial functional dressing [22]. The research of Wunsch et al. showed that collagen antibacterial functional dressing enhanced the phagocytic function of wound macrophages and reduced the inflammatory response of patients with breast cancer [23].

In addition, the experimental group has significantly lower levels of inflammatory factors after discharge, indicating that the collagen antibacterial functional dressing yields strong local anti-inflammatory and moisturizing effects to boost the growth of epidermal cells and promote metabolism.

The current study found that the skin-tingling sensation score of the patient was slightly lower in the experimental group. The reason may be ascribed to the individual differences between the patients. Also, continuous care ensured a high home care quality and resulted in a better recovery of the patients in the experimental group. A prior study has revealed that collagen antibacterial functional dressing contributed to the repair of skin defects in diabetic patients and promoted vascular regeneration [24]. Thus, collagen antibacterial functional dressing could also accelerate wound repair and reduce the pain of the patient with lower extremity skin injuries. Kasugai et al. treated patients with septic shock with collagen antibacterial functional dressing and compared them with Kanghuier's enhanced transparent paste. It was found that collagen antibacterial functional dressing facilitated vascular regeneration, reduced local edema, and relieved the stimulation of peripheral nerves by active factors after drug extravasation [25].

## 5. Conclusions

Collagen antibacterial functional dressing plus continuous care improves the local skin condition of patients with septic shock receiving norepinephrine, regulates the levels of inflammatory factors, reduces the risk of skin injuries, and enhances care satisfaction.

## Figures and Tables

**Figure 1:** Comparison of recovery time of patients with lower extremity skin injury, ^*∗∗∗*^*P* < 0.001.

**Table 1:** Comparison of the general information.

	Experimental group	Control group	*χ*2/*t*	*P*
*n*	60	60		
Gender (male/female)	41/19	42/18	0.039	0.843
Age (years)	50.11 ± 2.15	50.23 ± 2.16	0.305	0.761
Weight (kg)	56.21 ± 2.01	56.25 ± 2.10	0.107	0.915
BMI (kg/m2)	22.10 ± 2.10	22.12 ± 2.14	0.052	0.959
Primary disease				
AOSC	12	11	0.054	0.817
ALP	10	11	0.058	0.810
CRI	12	13	0.051	0.822
PC	8	7	0.076	0.783
ANP	10	11	0.058	0.810
COPD	8	7	0.076	0.783

AOSC: acute obstructive suppurative cholangitis, ALP: acute lobar pneumonia, CRI: chronic renal insufficiency, PC: posthepatitic cirrhosis, ANP: acute necrotizing pancreatitis, and COPD: chronic obstructive pulmonary disease.

**Table 2:** Comparison of skin sensation scores ($\bar{x}\pm s$, points).

	Burning		Itchiness		Stretching		Stinging	
	Before	1 month after	Before	1 month after	Before	1 month after	Before	1 month after
Experimental group	0.60 ± 0.08	0.34 ± 0.02	0.79 ± 0.06	0.45 ± 0.04	0.29 ± 0.04	0.15 ± 0.03	1.21 ± 0.05	0.78 ± 0.04
Control group	0.74 ± 0.05	0.49 ± 0.05	0.90 ± 0.08	0.65 ± 0.06	0.39 ± 0.05	0.26 ± 0.04	1.40 ± 0.06	1.00 ± 0.04
*t*	11.50	21.58	8.52	21.48	12.10	17.04	18.84	30.13
*P*	<0.001	<0.001	<0.001	<0.001	<0.001	<0.001	<0.001	<0.001

**Table 3:** Comparison of the incidence rate of skin injury of the lower extremities.

	*n*	Skin injury	No skin injury
Experimental group	60	3	57
Control group	60	14	46
*χ*2		8.292	
*P*		0.004	

**Table 4:** Comparison of the levels of inflammatory factors ($\bar{x}\pm s$).

	CRP (mg/L)		PCT (ng/L)		TNF-*α* (pg/mL)	
	Before	1 month after	Before	1 month after	Before	1 month after
Experimental group	172.65 ± 24.11	10.20 ± 1.21	25.56 ± 3.21	1.01 ± 0.25	20.12 ± 2.65	3.58 ± 1.20
Control group	172.56 ± 25.13	13.58 ± 2.23	26.14 ± 3.20	1.45 ± 0.30	20.23 ± 2.10	5.24 ± 2.15
*t*	0.006	2.503	0.285	2.354	0.079	1.273
*P*	0.996	0.024	0.778	0.033	0.938	0.222

**Table 5:** Comparison of care satisfaction rate (*n* (%)).

	*n*	Highly satisfied	Satisfied	Dissatisfied	Satisfaction rate
Experimental group	60	30 (50.0)	18 (30.0)	2 (3.3)	58 (96.7)
Control group	60	18 (30.0)	30 (50.0)	12 (20.0)	48 (80.0)
*χ*2					8.086
*P*					0.004

## Data Availability

The data can be obtained from the corresponding author upon reasonable request.
